RETRACTED

# Nursing of Gastrointestinal Peristalsis Function Recovery after Abdominal Mirror Surgery for Rectal Cancer Patients Based on Intelligent Electronic Medicine

**DOI:** 10.1155/2021/6668885

**Published:** 2021-04-22

**Authors:** Yanyan Ding, Sujuan Zhu, Jieqiong Pang, Zhitao Li, Congkun Ming, Xiaofang Song

**Affiliations:** ^1^Gastrointestinal Surgery Department, The Second People's Hospital of Dongying, Dongying 257335, Shandong, China; ^2^General Surgery Department, The Second People's Hospital of Dongying, Dongying 257335, Shandong, China; ^3^Department of Gastroenterology, The Second People's Hospital of Dongying, Dongying 257335, Shandong, China

## Abstract

In recent years, with the rapid development of colorectal surgery technology and laparoscopic instruments, laparoscopic radical resection of colorectal cancer has been widely used. Although laparoscopic surgery has the characteristics of small trauma, less blood loss, less hospitalization days, and low incidence of adverse reactions such as incision infection, it is still inevitable to have different degrees of gastrointestinal dysfunction after surgery. This paper mainly studies the recovery nursing of gastrointestinal peristalsis after abdominal mirror in rectal cancer patients based on intelligent electronic medicine. In this paper, an intelligent medical monitoring system is designed for the posterior care of rectal cancer patients with abdominal mirror image, which can realize the collection and transmission of wireless sign parameters of postoperative rectal cancer patients and improve the efficiency of postoperative monitoring in medical work. All parameter data are sent to the Lora base station in real time via Lora wireless communication, which is then uploaded to the medical monitoring platform. The experimental results showed that the first postoperative exhaust time of the treatment group using the intelligent medical monitoring system was significantly shortened, and the difference was statistically significant (*P* < 0.05). The first defecation time was shortened, and the difference was statistically significant (*P* < 0.05). The recovery time of total fluid diet was shortened, and the difference was statistically significant (*P* < 0.05). The above results indicate that the intelligent medical monitoring device designed in this paper has positive significance for improving the work efficiency of the hospital, the clinical experience of patients after abdominal mirror surgery for rectal cancer, and the real-time monitoring of signs of patients in intensive care.

## 1. Introduction

The recovery of gastrointestinal function after operation is an important aspect of rectal cancer after laparoscopic surgery and even the whole abdominal surgery. During this period, patients are affected by the disease itself, anesthesia, surgery, and other comprehensive factors, which easily lead to the disorder of multiorgan systems such as psychological, immune, and endocrine disorders and affect the postoperative recovery of gastrointestinal function [1]. Clinically, there are also many measures to promote the recovery of gastrointestinal function in this period, including perianaesthesia drugs, treatment intervention, early enteral nutrition and intestinal environment improvement, the use of gastrointestinal motility drugs, and exploration of gastrointestinal electrical stimulation [2]. There are also some comprehensive treatments of traditional Chinese medicine to promote the recovery of gastrointestinal function, such as oral administration, acupuncture, pedicure, acupoint application, ear acupoints, enema, and hot and electric hot compresses of Chinese medicine for external use; with the concept of prevention, treatment, and rehabilitation, integrated traditional Chinese and Western medicine intervention measures including physical therapy, psychological intervention, oral care, dietary posture guidance, postoperative function recovery exercise-integrated nursing intervention, and other multidisciplinary interventions jointly promote postoperative gastrointestinal function recovery. The intelligent medical monitoring system can provide users with real-time monitoring of signs and parameters [3]. It can not only be used for severe patients but also provide sign monitoring for patients who have just completed surgery and remote sign monitoring for the elderly at home who are unable to move.

RETRACTED

At present, the research of intelligent medical monitoring is a hot spot, and all countries in the world are paying close attention to medical monitoring. Wolf believes that traditional medical monitoring systems could be transformed into smart medical monitoring devices, equipped with sensors, to help patients become part of the diagnosis and treatment process. However, he did not make an empirical study [4]. Abdel proposed a framework for the detection and observation of type 2 diabetes based on computer-assisted diagnosis and the Internet of things [5]. The framework aims to obtain more data through the Internet of Things system to obtain a higher medical diagnostic accuracy. Experimental results also show the effectiveness and robustness of the algorithm. However, this system is only for preoperative diagnosis and does not involve postoperative nursing content [6]. Xiao has designed and developed a complete intelligent mobile-assisted healthcare architecture that provides medical feedback to patients via mobile devices by deploying biomedical and environmental data collected by sensors [7], but he did not experiment with this system.

RETRACTED

The intelligent medical monitoring system studied in this project can calculate the required signs parameters in combination with the signal collected by the sensor and then realize the real-time monitoring of the patient, including the patient's heart rate, blood oxygen, body temperature, and blood pressure. The data collected in real time can be displayed on the interface of the medical monitoring platform developed by the system. It has positive significance for improving hospital medical efficiency, physiological monitoring, and health management of patients with rectal cancer after laparoscopic surgery. It can effectively promote the recovery of gastrointestinal peristalsis after laparoscopic surgery in rectal cancer patients.

## 2. Application of Intelligent Medical Monitoring Device in the Nursing of Rectal Cancer Patients after Laparoscopic Surgery

### 2.1. Laparoscopic Gastrointestinal Surgery

#### 2.1.1. Characteristics of Laparoscopic Surgery

Laparoscopic surgery has small trauma, quicker recovery of intestinal function, less intraoperative complications, light postoperative pain, small body's immune disturbance, the advantages of rapid recovery, shorter hospitalization time, laparoscopic amplification effect at the same time, and clear field of vision and will not damage the surrounding tissue organs. Laparoscopic surgery has the advantages of low incidence of incisional hernia and beautiful incision [8, 9]. In recent years, laparoscopy is a minimally invasive technique, has been widely used in the operation in all the subjects, and has achieved very considerable success; gastrointestinal surgery is of no exception to the direction of minimally invasive, and studies have shown that laparoscopic surgery in the treatment of gastrointestinal surgery showed good effect, but, because of the large trauma of gastrointestinal tumors with carbon dioxide pneumoperitoneum, operation, and anesthesia, postoperative gastrointestinal dysfunction is seen, with even intestinal obstruction and other serious complications, so to promote the recovery of gastrointestinal function, reducing the incidence rate of complications is the key to improve the curative effect of patients.

#### 2.1.2. Gastrointestinal Dysfunction after Laparoscopic Surgery

Sympathetic nervous system diseases, parasympathetic nervous system diseases, and decreased gastrin secretion often occur after laparoscopic gastrointestinal surgery. At the same time, many factors such as physical injury during surgery, anesthesia, pneumoperitoneum, and internal organ strains caused by surgical instruments will slow down the recovery of surgery, and with the increase of inflammatory mediators, various disorders of gastrointestinal function will appear; common gastrointestinal functional disorders are exhaust bowel disorders, nausea and vomiting, abdominal pain, abdominal distension, etc. If the treatment is not appropriate or not in time, it will result in serious complications such as gastrointestinal obstruction, gastric retention, intestinal adhesion, and gastroparesis. Patients not only have to endure physiological pain but also have to bear the burden of costs caused by the increase in postoperative recovery time. Studies have shown that the incidence of gastrointestinal dysfunction after gastrointestinal surgery is 15%–40%, among which the incidence after pancreatoduodenectomy is relatively high, up to 20%–50% [12]. It is the common goal of clinical medical staff and scientific researchers to find simple, effective, and safe measures to promote the recovery of gastrointestinal function as soon as possible after gastrointestinal surgery.

RETRACTED

#### 2.1.3. Postoperative Gastrointestinal Dysfunction in Modern Medicine Treatment

The recovery of gastrointestinal function after surgery is a key link for the recovery state after surgery. Gastrointestinal function disorder is caused by many factors, and treatment should be carried out from many aspects. During abdominal surgery, the duration of intestinal exposure, wound reduction, and abdominal cavity flushing should be shortened as much as possible. Early treatment should strengthen nutritional support and timely supplement of electrolytes and trace elements [13]. According to traditional ideas, postoperative high potassium level in 2-3 days is easy to be caused by postoperative reasons such as large extracellular transfer of potassium, low urine volume, and blood transfusion. However, recent studies have found that preoperative fasting and intraoperative and postoperative potassium loss are prone to hypokalemia, and appropriate supplementation should be performed even if the serum potassium level is normal [14]. At present, the main drugs to improve gastrointestinal function in abdominal surgery are to promote gastrointestinal smooth muscle contraction.

*(1) Serotonin Receptor Agonist 4 (5-HT4)*. 5-Hydroxy tryptamine (5-HT) receptor is widely found in central and peripheral neurons. During human body movement, lumen chromaffin cells secrete a large number of serotonin agonists. Serotonin agonists in turn stimulate the intestinal wall between the 5a acetyl choline plexus to release serotonin receptors; serotonin agonists 4 can selectively stimulate chemical feelings trigger zone and vagus, play a dual role of inhibition of central and peripheral, and can promote gastrointestinal smooth muscle movement, so the serotonin is the best choice for the treatment of postoperative gastrointestinal disorders. The main action site of Cisapil is the digestive tract. The mechanism of action is to stimulate the 5-HT receptor and release ACh in the intestinal muscularis plexus, which can significantly improve esophageal, gastric, and duodenal reflux and enhance the large intestine and small intestine peristalsis. It is currently only an effective gastric stimulant for pseudoileus and can be taken for a long time [15].

*(2) Dopamine Receptor Antagonists*. Dopamine receptor antagonist mainly exerts antagonistic effect on the second receptor of dopamine, blocks the inhibition of dopamine on the gastrointestinal smooth muscle, relatively enhances the effect of acetylcholine on the smooth muscle, and then promotes the gastrointestinal peristalsis. The commonly used clinical drugs are methoxy clopramine and domperidone. Metoclopramine mainly acts on the upper digestive tract, has a central antiemetic effect and peripheral antagonistic dopamine effect, and can effectively promote the recovery of gastrointestinal function and reduce abdominal distension and abdominal pain [16]. Domperidone is a peripheral dopamine receptor antagonist, which can promote gastric contraction and duodenal peristalsis. Domperidone cannot pass the blood-brain barrier and thus reduces the occurrence of a series of reactions in vitro. However, metoclopramide can pass the blood-brain barrier, and a series of vertebral in vitro reactions such as delayed dyskinesia, ataxia, and Parkinson's syndrome are easy to occur in long-term use.

*(3) Motilin Receptor Agonist*. Erythromycin, a common macrolide antibiotic, is also a nonpeptide motilin receptor agonist, also known as Motilide, due to its similarity in molecular spatial structure to motilin. The mechanism of promoting gastrointestinal motility is to induce MMC contraction, and different doses directly affect the promotion effect. Large dose use can easily cause severe smooth muscle contraction, resulting in nausea, vomiting, and other adverse reactions of digestive tract. Studies have found that both erythromycin and motilin have similar structures, which can directly act on motilin receptors, release motilin and acetylcholine, and excite gastrointestinal smooth muscles [17, 18]. It has a significant effect on improving gastrointestinal motility, promoting gastric empty-out, eliminating nausea and vomiting, and shortening the length of hospital stay in premature infants. However, erythromycin may cause abnormal action potential in myocardium and increase the incidence of arrhythmia. Other macrolide derivatives, such as cefazolin, SK-506, and EM523, have the effect of promoting the gastrointestinal moment.

RETRACTED

### 2.2. Intelligent Medical Monitoring System

The intelligent medical monitoring system is mainly applied to postoperative patients, intensive care patients, and patients with chronic diseases [19]. It can continuously measure vital sign parameters such as heart rate, blood oxygen, body temperature, and blood pressure, so as to carry out efficient monitoring and auxiliary treatment for patients [20, 21]. The whole system is characterized by small size, complete functions, and portability. Based on Lora wireless communication technology, the monitoring distance is further and the network coverage is wider [22, 23].  Figure 1 shows the overall framework of the intelligent medical monitoring system. It is composed of blood pressure monitoring module, physical signs monitoring module, Lora base station, and medical monitoring platform.

#### 2.2.1. Continuous Blood Pressure Monitoring Module

Blood pressure is one of the physical signs of cardiovascular health and also a measure of an individual. We usually refer to blood pressure as arterial pressure. At present, the measurement method of blood pressure still cannot get rid of the restraint of the inflatable cuff. During the measurement process, the inflatable pressure and air release will bring great discomfort to patients, and the blood pressure value can only be measured at a certain moment [24]. The blood pressure monitoring module designed in this paper can well solve the above problems and can realize continuous blood pressure monitoring function. Its specific functions are as follows:

1. Signal acquisition and processing. Two pulse signals are collected by selecting appropriate photoelectric sensors at different positions and filtered, amplified, and sampled by the conditioning circuit [25]. Then, the blood pressure value of the measured object is calculated by the blood pressure algorithm. This method can get rid of the cuff and achieve continuous blood pressure measurement.
2. Real-time display function. In order for medical staff, patients, or patients' family members to grasp real-time information simply and intuitively, OLED display screen will be used to display the data in real time, and the display content is the blood pressure value of the tested object.
3. Alarm prompt. It is normal that the blood pressure value of human body will fluctuate due to the changes in external conditions and their own conditions. However, when there is a large fluctuation, it indicates that the body has lesions. Therefore, a large threshold can be set, and when there is a large fluctuation, an alarm will be automatically given to remind patients and medical staff.
4. Data communication. In this design, wireless Lora communication is adopted as the transmission medium between the hardware collection end and the medical monitoring platform, and the data frame format is developed to transmit the blood pressure data after processing and calculation to the PC end of the nurse station for display.

RETRACTED

#### 2.2.2. Sign Parameter Monitoring Module

The physical signs monitoring module integrates the real-time monitoring functions of heart rate, blood oxygen, and body temperature. At present, most of the monitoring tasks in hospitals are completed by various sign monitors. Meanwhile, nurses are required to make regular rounds of wards to understand the physiological status of patients, and the changes in various signs parameters of patients cannot be grasped in real time [26, 27]. The system collects all kinds of signals required by the sensor acquisition module, and then, the main controller calculates all signs parameters through a specific algorithm. Lora wireless communication technology is used to transmit the parameter information to the medical monitoring platform. The functions involved in this module are as follows:

1. Signal processing. According to the characteristics and generating mechanism of PPG signal, the sensor is used to collect the PPG signal at the fingertip. PPG signal belongs to low-frequency weak signal and is vulnerable to noise interference, so it needs circuit conditioning, which includes signal inversion, amplification, and filtering.
2. Alarm prompt. A buzzer is added to the circuit design to warn patients and medical staff automatically when signs and parameters fluctuate greatly.
3. Real-time display function. In order to grasp the monitoring information simply and intuitively, medical staff, patients, or their family members can increase the OLED display function to display the heart rate, blood oxygen saturation, and body temperature of the tested object.
4. Data communication. The design adopts wireless Lora technology to transmit the calculated physical sign parameters to the medical monitoring platform for display.

#### 2.2.3. Demand for Intelligent Medical Monitoring Platform

The medical monitoring platform, namely, the PC terminal of nurse station, as the terminal of vital sign parameter monitoring system, can receive, display, and manage the received data in real time. The analysis of each module is as follows:

1. Information management. Support the patient's personal information storage, including the information of bed number, name, gender, nursing level, age, contact information, medical condition introduction, and various monitoring data.
2. Real-time monitoring of physical sign parameters. As the main function module, this module can monitor the physiological parameter information of all patients in the whole department after successful login and also operate on patients in any bed in this department.
3. Data management. Store the bed number of each patient, along with information on blood pressure, temperature, heart rate, and oxygen, and support the patient's historical signs parameter data query. Real-time monitor data can be saved as a named date. In the later stage, users can select a record to view specific historical data, which has the role of adjuvant therapy.
4. User management. The system users are divided into superusers and ordinary users. Superusers can manage the information and permissions of ordinary users, while ordinary users can only manage patient data in their department. The system provides precise and fuzzy word query, and by entering a word of a patient's name on the home page, all information including the patient's name and bed number can be retrieved.

RETRACTED

### 2.3. Continuous Blood Pressure Measurement Algorithm

#### 2.3.1. Pulse Wave Conduction Time Method

Pulse wave conduction time (PTE) is a noninvasive method to detect blood volume change in arterial vessels by a photoelectric sensor. It uses the principle of light transmission or reflection. When the incident light is illuminated on the surface of the human body, the absorptive capacity of human tissues, muscles, bones, and blood to light is different, while the absorptive capacity of the same tissue is fixed and will not change with the light intensity [28]. According to Lambert–Beer's law,

(1) $$\begin{array}{c} \log\left(\frac{I_{0}}{I}\varepsilon \cdot C\cdot l\right). \end{array}$$

PPG signal acquisition principle: when light is irradiated to human tissues, the absorption of light by muscles, skin, bones, fat, water, and venous blood remains unchanged. However, the change in blood volume in the arterial blood tube will be caused by the beating of the heart, and the change in blood flow makes the absorption of light also present periodic changes [29]. Arterial blood constant component, venous blood, muscle, and bone have constant light absorption, so dc component is present at the receiving end, while AC component reflects the change in arterial tube volume. Therefore, light strength and small at the receiving end can reflect the beating situation of the heart [30].

The pulse wave transit time can calculate blood pressure because it can get rid of the restraint of the cuff and improve the comfort of the subject. The second reason is that the hardware system equipment can be used without repeated inflation and deflation. The most critical point is that for critically ill patients, continuous blood pressure measurement and continuous blood pressure value recording can be achieved [31].

RETRACTED

#### 2.3.2. Relationship between Pulse Wave Conduction Time and Arterial Blood Pressure

Pulse wave conduction time can be obtained indirectly through pulse wave propagation velocity. The formula of wave propagation velocity in an elastic tube is as follows:

(2) $$\begin{array}{c} c=\sqrt{\frac{Eh}{\rho D}}, \end{array}$$

where *E* is the elastic modulus, *h* is the thickness of vessel wall, *I*_*s*_ is the fluid density, and *D* is the inner diameter of the elastic tube at equilibrium.

There is an exponential relationship between the elastic modulus and the vessel cross-wall pressure [32], and thus, the following relationship is proposed:

(3) $$\begin{array}{c} E=E_{0}\cdot e^{rp}. \end{array}$$

The wave velocity formula is

(4) $$\begin{array}{c} c=k\sqrt{\frac{Eh}{\rho D}}. \end{array}$$

Pulse wave conduction time (PTT or PWTT) refers to the time taken for pulse waves to travel from one point to another during the transmission process in the arterial blood vessels. When the propagation distance is fixed, the pulse wave propagation velocity and pulse wave conduction time are related as follows:

(5) $$\begin{array}{c} C\frac{s}{T}. \end{array}$$

By substituting formulas (4) and (5) into formula (3), we can get

(6) $$\begin{array}{c} P=\frac{1}{\gamma }\left[\ln\left(\frac{\rho \text{ d}s^{2}}{aE_{0}}\right)-2\;\ln\;T\right]. \end{array}$$

As the heart beats, blood will periodically rush into the arterial tube, resulting in constant changes in blood pressure. During this process, the vessel wall will also have slight deformation. At this time, the changes in the inner diameter of the arterial wall and the thickness of the arterial wall can be ignored:

(7) $$\begin{array}{c} \frac{\text{d}P}{\text{d}T}=-\frac{2}{rT}, \end{array}$$

or

(8) $$\begin{array}{c} \Delta p=-\frac{2}{rT}\Delta T. \end{array}$$

According to the above formula, when vascular elasticity is ignored, blood pressure is linearly related to pulse wave conduction time. Therefore, the relationship between blood pressure and pulse wave conduction time can be simplified as follows:

(9) $$\begin{array}{c} P=a+b*PTT. \end{array}$$

In the formula, *a* and *b* are undetermined coefficients, reflecting the characteristics of individual arteries and vessels, which will change due to changes in vascular elasticity. However, in the short term, individual *a* and *b* values are fixed.

RETRACTED

## 3. Experimental Method of Intelligent Medical Monitoring Device

### 3.1. Source and Grouping of Cases

All the cases studied in this study were from patients undergoing laparoscopic radical resection of colorectal cancer in our hospital. The collection time was in the last year. The total number of samples studied in this study was 90 cases, including 30 cases in the treatment group and 30 cases in the two control groups. Among them, the treatment group adopted the intelligent medical monitoring system, the control group 1 adopted the hospital medical monitoring system, and the control group 2 adopted the traditional monitoring mode.

In this paper, a medical monitoring system was designed to provide postoperative care for patients undergoing laparoscopic radical resection of rectal cancer in our hospital. Cases were collected from patients undergoing laparoscopic radical resection of rectal cancer in our hospital in the last year. The total number of samples studied in this paper was 90 cases, including 30 cases in the treatment group and 30 cases in the two control groups. Among them, the treatment group adopted the intelligent medical monitoring system, the control group 1 adopted the hospital medical monitoring system, and the control group 2 adopted the traditional monitoring mode. As shown in Table 1, the basic data of the patients participating in the experiment are presented. The ratio of male to female was 17 : 13, 16 : 14, and 16 : 14. The age of the subject was approximately 60 years old.

### 3.2. Main Efficacy Indicators

The main efficacy indicators are as follows. laboratory examination results: preoperative and postoperative WBC, Hb, and PLT count data on the 1st and 3rd days; nutritional indicators: transferrin, albumin, and prealbumin; postoperative gastrointestinal function recovery time: including postoperative first exhaust time and postoperative first defecation time; restore full flow diet and half flow diet; abdominal distension, nausea, and vomiting and other gastrointestinal symptoms; gastrointestinal function score before and 7 days after operation; and VAS pain score before and 7 days after surgery (or until the day of discharge).

### 3.3. Experimental Operation Flow

The blood collection time points of each group were 2 fasting blood samples (lithium heparin tube, red anticoagulant tube, and 3 ml blood each) at 7 am before and 1, 3, and 7 days after surgery, respectively. After blood collection, the samples were placed in a 5°C refrigerator and centrifuged at a 5°C centrifuge at 3000 r/min for 15 min within 48 hours, and the supernatant was retained in a sterile 1.0 mL centrifuge tube. The samples were sealed and stored in a −80°C refrigerator for testing.

RETRACTED

## 4. Comparison of Experimental Data of Intelligent Medical Monitoring Equipment

### 4.1. Postoperative Initial Exhaust Time

In this paper, the postoperative first exhaust time of patients was counted, and the maximum, minimum, and median of the first exhaust time of patients in three groups were selected.

As shown in Table 2 and Figure 2, the difference in initial postoperative exhaust time among the three groups was statistically significant (*P* < 0.05). The LSD test was used for comparison between the two groups: compared with control group 2, the initial postoperative exhaust time of the first two groups was significantly shortened, and the difference was statistically significant (*P* < 0.05). Compared with the control group 1, the first postoperative exhaust time in the treatment group was shortened, and the difference was statistically significant (*P* < 0.05).

### 4.2. Time of Postoperative First Defecation

Similar to the statistics of the patients' first postoperative exhaust time, the maximum, minimum, and median of the first defecation time of the three groups of patients were still selected.

As shown in Table 3 and Figure 3, the difference in the first postoperative exhaust time among the three groups was statistically significant (*P* < 0.05). The LSD test was used for comparison between the two groups: compared with the control group 2, the first postoperative bowel movement time of the other two groups was shortened, and the difference was statistically significant (*P* < 0.05). Compared with the control group 1, the time of first postoperative defecation in the treatment group was shortened, with statistically significant difference (*P* < 0.05).

### 4.3. Postoperative Recovery Time of Whole Liquid Food

Similar to the previous two statistical indicators of patients, the maximum, minimum, and median values of postoperative total fluid recovery time of patients in the three groups were still selected.

As shown in Table 4 and Figure 4, the postoperative recovery time of total fluid diet of the three groups was statistically significant (*P* < 0.05). The LSD test was used for comparison between the two groups: compared with control group 2, the recovery time of all-liquid diet in the other two groups was shortened, and the difference was statistically significant (*P* < 0.05). Compared with the control group 1, the recovery time of patients in the treatment group was shortened, and the difference was not statistically significant (*P* < 0.05).

### 4.4. NRS Score 7 Days after Surgery

In this paper, the NRS scores of the three groups of patients at 7 days after surgery were counted, and the NRS scores of the first, third, fifth, and seventh days were selected, respectively.

RETRACTED

As shown in Table 5 and Figure 5, NRS scores of the three groups were compared 7 days after surgery, and the difference was statistically significant (*P* < 0.05). The LSD test was used for comparison between the two groups: compared with the control group 2, the NRS scores of the other two groups 7 days after surgery were lower than the control group, and the difference was statistically significant (*P* < 0.05). Compared with the control group 1, the NRS score 7 days after surgery was lower in the treatment group, and the difference was statistically significant (*P* < 0.05).

### 4.5. Postoperative Gastrointestinal Function Score Comparison

#### 4.5.1. Comparison of Postoperative Gastrointestinal Adverse Reactions

As shown in Table 6 and Figure 6, the comparison results of gastrointestinal adverse reactions 3 days after operation in the three groups were listed. In the treatment group, nausea occurred in 4 cases, vomiting in 3 cases, and abdominal distension in 5 cases. In control group 1, there were 8 cases of nausea, 6 cases of vomiting, and 6 cases of abdominal distension. In control group 2, there were 13 cases of nausea, 11 cases of vomiting, and 10 cases of abdominal distension. Statistical results showed that *P* < 0.05, and the difference was statistically significant.

#### 4.5.2. Postoperative Gastrointestinal Function Score Comparison

As shown in Figure 7, postoperative gastrointestinal function scores of the three groups were compared, and the difference was statistically significant (*P* < 0.05). It can be seen that the difference in gastrointestinal function scores between the control group 1 and the control group 2 in the first three days after the surgery was not significant. Three days after the surgery, the gastrointestinal function scores of the patients in the control group 1 gradually approached that of the treatment group on average, and the scores of the patients in the treatment group were all higher than those in the control group 1 and control group 2 within 7 days after the surgery.

## 5. Conclusions

With the rapid development of colorectal surgery techniques and laparoscopic instruments in recent years, laparoscopic radical resection of colorectal cancer has been widely used. Laparoscopic colorectal cancer surgery has the characteristics of less trauma, less blood loss, fewer days of hospitalization, incision infection, and low incidence of other adverse reactions. However, it is still inevitable to have different degrees of postoperative gastrointestinal dysfunction in clinic.

RETRACTED

In this paper, an intelligent medical monitoring system is designed and implemented, and its main functions are as follows: the front-end monitoring module combines Lora wireless communication to realize real-time monitoring of patients' blood pressure, heart rate, blood oxygen, and body temperature. The physical sign parameter monitoring module and the blood pressure monitoring module are responsible for the data collection and transmission, and the medical monitoring platform realizes the real-time display of all physical sign parameters as well as the management and storage of patient information. As can be seen from the test results, the intelligent medical monitoring system designed in this paper provides more efficient and convenient conditions for medical staff and is conducive to the recovery of gastrointestinal peristalsis function after abdominal mirror surgery for colorectal cancer patients and further explores the recovery of gastrointestinal peristalsis function after abdominal mirror surgery for colorectal cancer patients.

The intelligent medical monitoring system designed in this paper can basically meet the application requirements, but from the perspective of the long-term development of medical monitoring, the system still has the problem of continuous improvement. This system only realizes the monitoring of blood pressure, heart rate, blood oxygen, and body temperature. In the future, it can expand the monitoring of more signs and parameters so as to improve the monitoring needs of patients with different symptoms. Add the function of mobile phone monitoring software, so that medical staff can achieve mobile office in mobile phone terminal or PDA terminal. At the same time, patients and their families can access the monitoring data through the mobile phone and receive the doctor's advice to achieve more intelligent human-computer interaction.

## Figures and Tables

**Figure 1:** General block diagram of intelligent monitoring system.

**Figure 2:** The first exhaust time after operation in two groups.

**Figure 3:** Comparison of the first defecation time among the three groups.

**Figure 4:** The recovery time of full fluid diet in three groups after operation.

**Figure 5:** The NRS score of the three groups was 7 days after operation.

**Figure 6:** Comparison of postoperative gastrointestinal adverse reactions.

**Figure 7:** Comparison of postoperative gastrointestinal function scores.

**Table 1:** Basic information of patients.

Group	Sex ratio (male : female)	*N*	Age	Weight	Defecation (day)
Control group 1	17 : 13	30	61.8 ± 6.37	57.19 ± 7.24	2.14 ± 1.58
Control group 2	16 : 14	30	60.9 ± 6.25	59.36 ± 7.15	2.19 ± 1.38
Treatment group	16 : 14	30	60.4 ± 6.52	56.27 ± 7.06	2.27 ± 0.94

RETRACTED

**Table 2:** The first exhaust time after operation in three groups.

Group	Minimum	Median 1	Median 2	Median 3	Median 4	Maximum
Treatment group	18.97	20.07	20.12	20.34	20.41	21.34
Control group 1	20.38	21.97	22.08	22.19	22.31	23.95
Control group 2	24.12	25.43	25.57	25.68	25.71	26.97

**Table 3:** Comparison of the first defecation time among the three groups.

Group	Minimum	Median 1	Median 2	Median 3	Median 4	Maximum
Treatment group	24.83	26.47	26.62	26.83	26.95	28.79
Control group 1	27.21	28.41	28.49	28.64	28.81	30.40
Control group 2	29.53	31.07	31.05	31.38	31.53	33.06

**Table 4:** The recovery time of full fluid diet in three groups after operation.

Group	Minimum	Median 1	Median 2	Median 3	Median 4	Maximum
Treatment group	26.34	27.94	28.06	28.23	28.35	29.92
Control group 1	27.33	28.94	29.01	29.10	29.27	30.81
Control group 2	31.68	34.07	34.14	34.29	34.46	37.12

**Table 5:** The NRS score of the three groups was 7 days after operation.

Group	First day	Third day	Fifth day	Seventh day
Treatment group	4.62	3.46	2.74	1.47
Control group 1	5.14	3.90	3.06	1.84
Control group 2	5.91	4.63	3.57	2.27

**Table 6:** Comparison of postoperative gastrointestinal adverse reactions.

Group	Nausea	Vomiting	Abdominal distention
Treatment group	4	3	5
Control group 1	8	6	6
Control group 2	13	11	10

## Data Availability

No data were used to support this study.
